The article "miR-451 on Myocardial Ischemia-Reperfusion in Rats by Regulating AMPK Signaling Pathway" was retracted in 2024. Reasons: signs of a paper mill; compromised peer review; unreliable results or conclusions.

# miR-451 on Myocardial Ischemia-Reperfusion in Rats by Regulating AMPK Signaling Pathway

**DOI:** 10.1155/2021/9933998

**Published:** 2021-07-06

**Authors:** Yulin Guo, Jie Gao, Yan Liu, Xitao Zhang, Xiangguang An, Jian Zhou, Pixiong Su

**Affiliations:** Department of Cardiac Surgery, Beijing Chaoyang Hospital, Capital Medical University, Beijing 100020, China

## Abstract

Myocardial infarction is the main cause of death in patients with coronary heart disease. At present, the main method to treat cardiovascular disease is perfusion therapy. Myocardial ischemia-reperfusion will inevitably lead to reperfusion injury, which is also a major problem in the treatment of cardiovascular diseases. It has been reported that mir-451 in microRNA family participates in the protection of myocardial ischemia-reperfusion by regulating AMPK. The aim of this study was to investigate the effect of mir-451 on myocardial ischemia-reperfusion in rats by regulating AMPK signaling pathway. Sixty adult male rats were selected to establish myocardial ischemia-reperfusion animal model by ligating and loosening coronary artery. The expression level of mir-451 was regulated by injection of mir-451 virus vector and antibody, and the effect of increased or decreased mir-451 expression level on the activity of AMPK signaling pathway was detected. The myocardial infarct area and apoptosis rate of myocardial tissue were detected after 75 min ischemia-reperfusion. The results showed that when the expression level of mir-451 decreased by 15.7%, the activity index of AMPK signaling pathway was increased by 18.3%, the infarct area was reduced by 22.4%, and the apoptosis rate of myocardial cells was decreased by 25.2%. At the same time, the pathological structure of myocardial tissue was improved. Therefore, mir-451 is an inhibitor gene of AMPK signaling pathway. Reducing the expression of mir-451 can enhance the activity of AMPK signal pathway, and the increase of AMPK signal pathway activity is beneficial to reduce myocardial ischemia-reperfusion injury.

## 1. Introduction

Cardiovascular disease is one of the intractable diseases threatening human life and health in today's society. According to statistics, due to myocardial ischemia necrosis and vascular recanalization, it often induces ischemia-reperfusion injury, which in turn leads to heart failure (HF), causing myocardial high mortality from infarction.

Apoptosis is an important part of ischemia-reperfusion injury (I/R), and it mostly occurs in the early stage of I/R injury. miR-451 is abundantly expressed in myocardial tissues, and it has been found in researches in related fields that miR-451 can promote cell apoptosis [1]. Many recent studies have shown that the AMPK signaling pathway is related to ischemia-reperfusion injury in various organs. This signaling pathway is composed of a series of transmembrane receptors, corresponding ligands, modifier genes, and transcription factors and regulates cell proliferation and differentiation [2]. Studies have found that the AMPK signaling pathway plays a key role in inflammation and apoptosis caused by renal ischemia-reperfusion injury. Upregulating the expression of the key protease of AMPK signaling pathway myocardial adenylate-activated kinase through miR-451 can significantly reduce inflammatory factors. Expression reduces cell apoptosis, which is very important to reduce myocardial ischemia-reperfusion injury [3].

In order to explore the specific effects of miR-451 on myocardial ischemia-reperfusion in rats by regulating the AMPK signaling pathway, a large number of related materials were reviewed. Among them, Song et al. gave a detailed introduction to the role of microRNA in the human body and its family members, discussed its related mechanisms involved in body regulation, pointed out that there is a close relationship between microRNA genes and a variety of diseases, and studied the corresponding targets of microRNA genes which are the key to the treatment of many diseases [4]. In their article, Yu et al. introduced the role of myocardial adenylate-activated kinase AMPK in detail, pointed out that the myocardial adenylate-activated kinase AMPK is one of the important elements in human myocardial tissue, and explored the process and principle of AMPK inhibiting cardiomyocyte apoptosis [5]. Bujak et al. clearly pointed out in their article that miR-451, as a noncoding RNA, can effectively enhance the activity of the AMPK signal in the pathway, emphasizing that the high level of miR-451 expression will inhibit the activity of the AMPK signal pathway, thereby exacerbating myocardial ischemia and reperfusion [6]. Wen et al. introduced the mechanism of myocardial ischemia-reperfusion injury, they pointed out that although reperfusion therapy can treat a variety of vascular diseases, it is very easy to cause reperfusion injury; they emphasized that there is no good treatment for reperfusion injury [7]. Zhenwei et al. found through research that miR-451 has a profound effect on myocardial ischemia and reperfusion by continuously inhibiting its active expression in AMPK signaling pathway; this mechanism is applicable to all cardiovascular diseases, while emphasizing that the role of miR-451 in the myocardial tissue is just the opposite [8].

As a new type of nanomaterial, ceria nanoparticles have the characteristics of relatively small particle size and large surface area, so there are more oxygen vacancies on the surface [9]. This feature makes it easier to take part in the redox process, which has a certain potential for scavenging regenerative free radicals. It can directly scavenge O_2_, Ho, and other free radicals; can avoid cell injury caused by lipid peroxidation and free radical reaction; and has antioxidation, anti-inflammatory, and antiapoptotic effects. Nrf2 is an important gene controlled by oxidative stress. The antioxidant response elements in the upstream promoter region of antioxidant genes combine with Nrf2 to induce the expression of a series of endogenous antioxidant proteins, antioxidant protective enzymes, and anti-inflammatory and other cellular genes. For example, it regulates the expression of quinone oxidoreductase and heme oxygenase to maintain the cell's oxidative and antioxidant balance [10]. Nanoceria pretreatment can upregulate the expression of Nrf2 in reperfusion myocardium, increase the expression of downstream cell protective genes NQO1 and HO-1, reduce the oxidative damage of reperfusion myocardium, and protect the myocardium.

Prussian blue nanoparticles (PBNPs) are chemically synthesized products with antioxidant capacity [11]. PBNPs can protect the cells from the influence of ultraviolet and lipopolysaccharide and protect the hippocampal cells from damage during reoxygenation. This suggests that PBNPs may be a potential protective agent against ischemia-reperfusion injury. PBNPs can mimic the ability of three antioxidant enzymes and have strong affinity for hydroxyl radicals. In the process of cell apoptosis, these abilities make PBNPs become a powerful ROS scavenger, reducing the oxidative stress injury and apoptosis of cells. PBNP pretreatment can improve the ability of oxygen free radical scavenging and antilipid peroxidation of cardiomyocytes and reduce the apoptosis of cardiomyocytes. So PBNPs have protective effect on myocardial ischemia-reperfusion injury.

Tissue factor plays a key role in the occurrence of ischemia-reperfusion injury. Tissue factor as a target, reducing its synthesis and release, can effectively prevent myocardial ischemia-reperfusion. Antisense oligodeoxynucleotides (AODN) can be used to block the transcription of tissue factor genes and have the advantages of strong specificity, good safety, and simple operation [12]. With the rapid development of biotechnology, physics, chemistry, and other fields, nanotechnology has begun to be more applied in the medical field. Polyamide amine dendrimer (PAMAM-D) nanocarriers are newly developed nanoscale gene transfer vectors that can be used to carry AODN for gene therapy.

In the study of the specific effects of miR-451 on myocardial ischemia-reperfusion in rats by regulating the AMPK signaling pathway, this article summarizes and analyzes the research experience and results of a large number of predecessors. In addition, this article has carried out some research on the research content and detection methods. The specific innovation has the following two points: First, this article uses the PCR detection method to measure the AMPK signal pathway activity and uses SSEC software system to collect and analyze the statistical data of rat myocardial ischemic area and apoptosis-related detection results, so as to be scientific and objective. Based on this, the relationship between miR-451 and myocardial adenylate-activated kinase AMP was discussed. Second, this model laboratory simulation is used to establish a model of inhibiting rat myocardial cell ischemia-reperfusion myocardial injury in the late stage, to explore the role of miR-451 in rat ischemia-reperfusion myocardial cell apoptosis, and to study how miR-451 can greatly enhance the activity of AMPK signaling pathway, thereby reducing myocardial ischemia-reperfusion injury and protecting the myocardium.

## 2. Myocardial Injury Mechanism and MicroRNA Action

### 2.1. Mechanism of Myocardial Ischemia-Reperfusion Myocardial Injury

When the ischemic acute myocardial bulb undergoes reperfusion, it is conducive to a series of adverse physiological events, such as acute arrhythmia, myocardial muscle contraction and vasodilation, and another cardiac dysfunction. This ischemia is mainly due to ischemic regenerative perfusion myocardial injury (I/R), myocardial infarction I/R (MIRI), which is a major cause of the prognosis of acute myocardial infarction [13]. During myocardial ischemia-regenerative perfusion, various rapid temperature changes may occur, which may aggravate myocardial damage and eventually lead to acute death of myocardial cells. The main pathological changes include increased blood oxygen free radicals (OFR), mucosal infiltration of inflammatory nodules, calcium overload, abnormal microcirculation, abnormal apoptosis, and abnormal metabolism of higher energy cells. Persistent acute myocardial ischemia can directly cause myocardial endometrial injury and endothelial cell death [14]. Early reperfusion can significantly reduce the severity of early myocardial ischemic tissue damage, but many of them have multiple reperfusions in the lung and through long-term clinical studies in animals. It has been observed that blood flow concentration in the myocardium can be effectively improved. But it will also increase myocardial damage caused by pure blood myocardial ischemia and infarction, arrhythmia, enlarged infarct ischemic area, persistent ischemia, acute ventricular contraction, and decreased lung function [15]. Changes in pathological structure may also lead to acute myocardial angioedema, loss or destruction of membranes and membranes of organs such as membranes and epithelial cell membranes, tissues with mild destruction or destruction, ultrastructural changes in muscles and fibers, and destruction of microvascular tissue without regeneration perfusion [16].

During ischemia-reperfusion, neutrophils are activated when they contact endothelial cells and then release some toxic inhibitors, such as antideoxy free radicals, proteases, elastin, and collagenase [17]. These toxins in human cells may destroy human endothelial connective cells, inhibit the expansion of physiological capillary walls and inhibit antithrombotic cell mechanisms, and may increase the permeability of human capillary walls. After reperfusion, the release of P-1-based selective cytokines (PSL), intercellular adhesion molecules (ICAM), and inflammatory adhesion mediators can directly lead to endothelial leukocyte vascular activation and mucosal adhesion and simultaneously produce a large amount of whether the EC expression of the superoxide anion cation and the superoxide anion cation receptor depends on the vascular arterioles. Interleukin 33 (il-33) has a good protective effect on cells [18]. Researchers found that il-33 can effectively upregulate the positive expression of p38 in cardiomyocyte cytokines, activate the signal transmission pathway in map, increase the expression ratio of bcl-2/BAX, reduce the positive expression of bcaspase-3, and reduce the expression level of other inflammatory response factors, so the treatment can reduce the area of myocardial infarction, can inhibit other inflammatory factors, and may reduce the apoptosis of myocardial cell nuclei [19]. Some clinical researchers have found that the two signal inhibition pathway devices of MAPK can effectively inhibit the transfer of rat nuclear activity factor f-kb (NF-kb) to the core of the rat nucleus and reduce the effect of the rat nucleus on the structure and nerve function of the heart and severe damage, thereby effectively protecting the rat myocardium.

After ischemia and reperfusion, the OFR reaction destroys the endothelial cells in the tiny blood vessels, resulting in vascular cell membrane damage, mitochondrial tissue dysfunction, endothelial cell protein synthesis and vasodilation response factor cell release, and the function of abnormal microvascular tissue. The permeability of the inner wall of vascular cells is greatly increased, and the increased edema of the intercellular membrane limits the normal expansion of local microvessels. Therefore, the local biological membrane cells are damaged due to the interaction between the membrane cell surface and local white blood cells. As the degree increases, white blood cells adhere to each other, leading to local capillary wall blockage [20]. Nitric oxide (NO) cannot only participate in the normal regulation of coronary arteries and cardiovascular relaxation but also play an important guiding role in the prognosis of chronic cardiomyopathy and the normal recovery of myocardial motor function after myocardial ischemia [21]. Transient coronary I/R damage caused by excessive arterial blood supply or cardiac dysfunction may weaken the coronary EC tube and produce. Neutrophils may play an important role in inhibiting acute myocardial ischemia-reperfusion [22]. Activating the neutrophil cytoplasmic receptor can release more than 30 kinds of neutral proteolytic enzymes at the same time, including neutral collagenase, elastin binding protein, metalloprotease, heparinase, and neutral serine binding protease, directly causing injury after infusion.

### 2.2. The Role of MicroRNA in Ischemia-Reperfusion Injury

In the continuous occurrence of various ischemic heart diseases and the development and evolution of the disease, the main predisposing factor of tissue cell damage is not due to ischemia itself but due to the inability to recover a large amount of blood supply, and free radical cells are overly attacked, and the recovery is due to tissue. Cells prevent a large amount of blood supply, causing secondary ischemic damage to various tissue cells [23]. Tissue cells are called cerebral ischemic regenerative perfusion or brain injury. Other damages that may be caused by ischemia-precellular perfusion are far greater than other damages that may be caused by cellular ischemia itself, such as insufficient blood oxygen supply and cellular oxidative stress [24]. It may directly lead to benign death of heart cells (including cell necrosis and apoptosis), hypertrophy, vascular thrombosis, fibrosis and cardiac dysfunction. MicroRNA is a kind of informal coding function RNA with length-regulated coding mechanism. They are widely distributed in eukaryotes; they are highly conserved in sequence and have tissue specificity. miRNA plays a negative regulatory role in the body [25]. Through the principle of base complementary pairing, miRNA specifically binds to target mRNA to induce a silencing complex, which can degrade target mRNA or inhibit the translation of target mRNA, thereby effectively regulating the level of main proteins and expression rates in human cell tissues. It refers to an endogenous level-regulating gene mechanism that is expressed on the genome containing horizontal movement-regulating enzymes after gene transcription [26]. miRNA is closely related to the early occurrence and development of a variety of brain diseases and especially plays a special role in cerebral ischemia regeneration and perfusion brain injury. The level of independent expression regulation of miRNA in vivo can be affected and regulated by many other factors, such as an independent expression regulation of primary cell transcription by cellular transcription inhibitors [27].

The most studied problem in human myocardial ischemic tissue is the relationship between myocardial miRNA and myocardial ischemia regenerative perfusion myocardial injury. A recent study showed that mir-123 is the most abundant and protective cell miRNA in cardiomyocytes. mir-133, mir-126, mir-214, mir-24, mir-454, mir-409, mir-125b, mir-144, and mir-451 together undergo multiple apoptosis after cardiomyocyte remodeling in the stage; it can play an important protective role. For example, mir-133, mir-204, mir-454, mir-409, and mir-125b can play the role of a variety of protective agents by cooperating with genes after myocardial apoptosis. Inhibition of benign apoptosis of cardiomyocytes and migration and inhibition of inflammatory metabolic reactions promote the formation of capillary walls [28]. Upregulating the expression of the parameter mir-133a in the acute myocardial cell expression of rats after the first ischemia-hypoxic perfusion myocardial injury can significantly effectively inhibit a large number of myocardial cell apoptosis, reduce the area of myocardial infarction in rats after reischemia-perfusion, and improve human. Some target cell genes of mir-454 may include not only target genes that promote apoptosis but also some target genes that resist apoptosis. The specific effect of the increased level of mir-494 cell expression in genetically modified mice allows it to effectively promote the normal recovery of myocardial cell immune function after myocardial ischemia and regeneration and perfusion and can inhibit a large number of cardiomyocytes and cell apoptosis. mir-126 and mir-220 can effectively promote the formation of malignant hemangioma [29]. The downregulation of the expression of mir-126 in mice may cause extensive acute vascular intimal defects, such as acute rupture of the vascular intimal. The significant downregulation of mir-280 expression under low oxygen concentration conditions will directly lead to the migration of the endothelial mesenchymal nuclei of coronary vascular cells and a significant decrease in the survival rate of vascular nuclei. mir-144 and mir-451 coordinately regulate the oxygenase 2 signal of the binding enzymes in CLB and CUG in the protein cycle as a pathway for transducing enzymes, so they have an important synergistic regulatory effect [30].

Studies have shown that the high normal expression of mir-201 can effectively inhibit the active proliferation, migration, and angiogenin production of bone marrow endothelial vascular cells by inhibiting the normal expression of RHOB in cells, which is lower than the normal downregulated mir-201. Its expression has the opposite inhibitory effect on it. At the same time, the results of gene silencing research in RHOB also clearly show that the benign proliferation of cortical leukocytes and the production of capillary walls in humans are severely damaged [31]. The mir-29 family, including mir-219a, mir-219b, and the entire mir-219c, is mainly expressed normally in fibroblasts of the entire heart and can regulate the normal expression of various genes related to the process of cardiac fibrosis, such as the heart, collagen, and the heart layer adhesion collagen. In experiments using the ischemia-regenerative perfusion method in vivo and in vitro, the obvious downregulation of mir-219 expression lies in the promotion of acute fibrous sclerosis of the myocardial wall by continuously inhibiting elastin collagen and inhibiting the repeated expression of elastin collagen [32]. In addition to the normal expression of molecular genes related to the cell fibrosis process, mir-219 also effectively regulates the normal expression of molecular genes related to the cell and apoptosis process. Studies have found that the expression of mir-29 is significantly downregulated after ischemia-reperfusion myocardial injury, which may lead to the upregulation of myeloid fibrotic leukemia 5 protein (an important member of the bcl-2 antiapoptotic protein family), thereby effectively inhibiting cell apoptosis and necrosis. However, the significant downregulation of mir-219 expression may lead to significant changes in the expression of myeloid fibrosis protein, which has a strong damage to the structural remodeling of fibrotic myocardial injury after ischemia-reperfusion.

## 3. Experiment of Polyethylene Wear Particles to Induce Osteolysis

### 3.1. Laboratory Animals and Related Equipment

In this experiment, 60 male rats were selected as experimental subjects, with an average age of 15 to 24 months and a weight of 260 ± 10.0 g. They were raised in separate cages according to the national standard sentinel feeding specifications. The rats were checked before the experiment health status, and mice with abnormal health were excluded. The rats were randomly divided into the operation control group, miR-451 upregulation observation group, and miR-451 downregulation observation group, with 20 rats in each group. The relevant equipment and reagents required for this experiment are shown in Table 1.

### 3.2. Creation of Myocardial Ischemia-Reperfusion Model

Rats were anesthetized by intraperitoneal injection of sodium pentobarbital (SOMG/kg). The limbs of the rat were fixed on the operating table with a rubber ring. The fixation should be firm, and the trachea should be intubated through the mouth. At the same time, care should be taken to avoid tracheal injury caused by rough operation during tracheal intubation. The success of tracheal intubation can be judged by observing whether the fluctuation of the rat's chest is consistent with the rhythm of the ventilator and whether the rat has hypoxia symptoms. The endotracheal tube was secured with a tape to prevent it from falling off. A small animal ventilator is connected through a flexible hose. The leads of the electrocardiograph were connected to the limbs of the rat. Observe the ECG waveform to determine if the leads are well connected. When the heartbeat is the most obvious, shave off hair, sterilize the incision with iodophor from the inside out, spread out the towel, open the chest layer by layer, gently pierce the pericardium with tweezers, adjust the chest opener appropriately to expose the heart, and take care of the round shape both ends of the needle and the needle holder, so as not to damage the surrounding tissues and organs. The ST segment of lead II increased significantly (increasing amplitude > 0.5 mV, ECG parameter setting, 18 mm/MV, and 20 mm/s), proving that the left anterior descending branch has been successfully ligated. After the ligation lasted for half an hour, the ligature was loosened and the ST segment of ECG lead II was significantly reduced, proving the successful reperfusion.

### 3.3. Regulate miR-451 Expression Level

Pre-mir-451/asmir-451 was chemically synthesized and digested at both ends of the microRNA with AGEI and ECORI and then ligated to the adenovirus solution expression vector linearized by strains AGEI and ECORI. Product cells were transformed into bacteria-competent cells. It was identified as a positive clone by colony PCR amplification, and then the positive clone target plasmid was sequenced and compared. The correct positive clone was sequenced and identified as successful. Target plasmid, which was amplified by colony PCR. After homologous recombination with the linearized skeleton plasmid in the target strain skeletal cell dh5a of Escherichia coli, colonies ad-mir-451 and colony ad-asmir-451 were formed in the strain dhek293 cells, respectively. After amplification and purification, the average titer of the adenovirus cell solution of this strain can meet the average titer requirements in vivo and in vitro obtained in vitro experiments. By injecting mir-451 vector virus into rats, the expression level of mir-451 increased. The expression level of mir-451 can be reduced by injecting mir-451 antibody into rats.

### 3.4. Measurement of Myocardial Infarction Area

After 5 hours of reperfusion, the rats were anesthetized. LAD was ligated in situ and 5 ml of 2.5% fluorescent blue pigment was injected through the jugular vein into the right ventricle. After removing the sliced heart from the left ventricle, the atrium and right ventricle were removed, rinsed with ice phosphate buffer, and frozen. The left ventricle is then cut into 1 mm thick transverse slices, and the right ventricle is placed in a 2% TTC solution (TTC dissolved in a buffer at 2% pH 6.4, concentration 0.4 mol/l) at 37°C. The blood region of the infarcted region (white and black region) of the ischemic region and the infarcted region (red region and black or white region) of the ischemic region are measured, and the ratio of the difference between the infarcted ischemic regions is measured: sliced and sliced ischemic infarct areas. The area was calculated to determine and assess the area of each myocardial infarction.

### 3.5. Cardiomyocyte Apoptosis Detection

Taking the above-mentioned cardiomyocytes after ischemia and reperfusion, add an appropriate amount of 0.65% trypsin to completely separate the cells, and at the same time, dilute the 30 × bind buffer with deionized water into 1 × binding buffer. Place the above-treated cells in a centrifuge tube at room temperature (5000 rpm/min, 10-18 min); after centrifugation, resuspend the cells with 1 × binbuffer cold solution, adjust the concentration to 1X106/ml, draw about 300 *μ*l of the above cell suspension, and place In the EP tube, drop 6 *μ*l, Annexin/FITC solution, and 10 *μ*l 20 mg/ml solution. Mix the lip solution, incubate at room temperature for 15 minutes in the dark, and then drop 400 *μ*l 1 × binding buffer into the test tube for flow cytometry analysis.

### 3.6. Observation of Pathological Structure of Myocardial Tissue

After perfusion, the rats were sacrificed, the heart was taken out, the left ventricular myocardium tissue was taken out after washing with saline, fixed in formaldehyde solution and hematoxylin and eosin staining solution, and paraffin-embedded sections were deparaffinized, moistened distilled water, and stained with water. After washing for 10 minutes, washing for 20 seconds, and staining the serum for 5 minutes, the filter paper was blotted dry, dehydrated with anhydrous ethanol 3 times, and then mounted. The pathological changes of the rat myocardial tissue were observed under a fluorescence microscope.

### 3.7. AMPK Signaling Pathway Activity Detection

The activity of the AMPK signaling pathway was detected by immunohistochemistry. The specific method is as follows. Add each aliquot of 30 mg of phosphorylated protein to the holes in the 92-well plate, and precoat each hole with the recombinant myosin phosphorylation target subunit (MYPT1). After 30 minutes of incubation at 200°C, the myocardial adenylate-activated kinase AMPK protein can phosphorylate the Thr896 site of MYPT1. Next, add 200 ml of peroxidase-conjugated anti-phosphor SM-PCR650 antibody and react at room temperature for 3 hours. The absorbance value of each well at 540 nm was measured on a microplate reader, and the activity level of AMPK signal pathway and the expression of myocardial adenylate-activated kinase AMPK were measured according to the standard curve and the obtained formula.

## 4. Experimental Results of miR-451 Regulating the AMPK Signaling Pathway on Myocardial Ischemia-Reperfusion in Rats

### 4.1. Analysis of the Effect of Adjusting the Expression of miR-451 on Cardiac Motility, AMPK Signaling Pathway Activity, and Myocardial Cell Apoptosis Rate

The results of the study showed that there was almost no significant difference in cardiac dynamics between the groups before reperfusion (*P* > 0.05). In addition, at the end of 30 minutes after a perfusion, in addition to the control group is the mir-451 upregulation group of the remaining control groups. Compared with the other mir-451 downregulation group and the basic value, lv-deep was significantly higher than the basic value (*P* < 0.05), and the basic values of HR, LVDP, and ±DP/dt were all significantly reduced (*P* < 0.05). Compared with the 451 upregulation group, LVEDP in the miR-451 downregulation group was significantly reduced (*P* < 0.05), and HR, LVDP, and ±DP/dt were significantly increased (*P* < 0.05). Compared with the control group, the miR-451 downregulation group was significantly higher in LVEDP (*P* < 0.05), and HR, LVDP, and ±DP/dt were significantly reduced (*P* < 0.05). This conclusion proves that the upregulation of miR-451 will lead to the decrease of left ventricular contractile function in rats and the upregulation of miR-451 expression. The relevant data of rat left ventricular hemodynamics after regulating the expression of miR-451 are shown in Table 2.

The results of the study showed that when the expression of miR-451 increased, the activity of the AMPK signaling pathway decreased and, when the expression of miR-451 decreased, the activity of the AMPK signaling pathway increased. When the expression level of miR-451 decreased by 15.7%, the activity index of AMPK signaling pathway increased by 18.3%, and when the expression level of miR-451 increased by 12.6%, the activity index of AMPK signaling pathway decreased by 19.5%. There were statistically significant differences between the AMPK signal pathway activities of the miR-451 upregulated group and miR-451 downregulated group and the control group (*P* < 0.05). With the prolongation of myocardial ischemia-reperfusion time, the amplitude of the AMPK signaling pathway activity index increased, and the increase in AMPK signaling pathway activity in the miR-451 downregulated group was lower than that of 12-hour perfusion. At the same time, the activation of adenylate in rat myocardium was detected. The increase in the expression of the kinase AMPK proves that the expression of the myocardial adenylate-activated kinase AMPK is directly proportional to the activity of the AMPK signaling pathway and miR-451 inhibits the activity of the AMPK signaling pathway. The results of the study show that downregulating the expression of miR-451 can increase the activity of AMPK signaling pathway. The relevant data are shown in Figure 1.

It can be seen from the data in Figure 1 that downregulating the expression of miR-451 can increase the activity of the AMPK signaling pathway. When the expression level of miR-451 decreases by 15.7%, the activity index of the AMPK signaling pathway increases by 18.3%.

Studies have shown that when the expression of miR-451 decreases, the apoptosis of rat cardiomyocytes will decrease, and when the expression level of miR-451 decreases by 15.7%, the apoptosis index of rat cardiomyocytes is (15.3 ± 2.36), and the expression level of miR-451 increases by 11.6%. The apoptotic index of rat cardiomyocytes at time was 21.4 ± 1.86. Comparing the results of clinical trials between the mir-451 downregulation group and the control group, the rapid apoptosis rate of cardiomyocytes was significantly lower than that of the control group. The AMPK signaling pathway reflected signals so that its pathway activity could be significantly reduced, and the rats were subjected to myocardial ischemia and reperfusion. When cardiomyocytes undergo rapid apoptosis, the expression level of miR-451 is directly proportional to cardiomyocyte apoptosis, and the expression of myocardial adenylate-activated kinase AMPK is inversely proportional to cardiomyocyte apoptosis. The research results show that miR-451 can effectively reduce the apoptosis rate of cardiomyocytes during ischemia-reperfusion by reducing the activity of AMPK signaling pathway. The relevant data are shown in Figure 2. It can be seen that miR-451 can effectively reduce the myocardial cell apoptosis rate during ischemia-reperfusion by reducing the activity of AMPK signaling pathway. The expression level of miR-451 is reduced by 15.7%, and the apoptosis rate of rat myocardial cells is reduced by 25.2. %.

### 4.2. Analysis of the Effect of miR-451 on Myocardial Ischemia-Reperfusion Injury in Rats by Reducing the Activity of AMPK Signaling Pathway

The results of the study showed that the miR-451 expression regulation observation group and the clinical control group comprehensively measured the left ventricular infarction area and ischemia risk area. Upregulating the expression of miR-451 reduces the activity of the AMPK signaling pathway. The myocardial infarct area increases after myocardial ischemia-reperfusion in rats and decreases the activity of the AMPK signaling pathway by downregulating the expression of miR-451. Compared with the results of the control group, there was a statistical difference (*P* < 0.05). The myocardial infarction area of rats in the control group was smaller than that in the miR-451 upregulated group and larger than that in the miR-451 downregulated group, indicating that AMPK signaling pathway activity and myocardial ischemia-reperfusion. The infarct size is inversely proportional, and the myocardial adenylate-activated kinase AMPK is involved in preventing the formation of thrombus in myocardial tissue. The results of the study show that miR-451 can reduce the area of myocardial infarction during myocardial ischemia-reperfusion in rats by reducing the activity of AMPK signaling pathway. The specific data are shown in Figure 3.

From the data in Figure 3, it can be seen that miR-451 can reduce the myocardial infarction area during myocardial ischemia-reperfusion in rats by reducing the activity of AMPK signaling pathway. When miR-451 expression level is reduced by 15.7%, the rat myocardial infarction area is reduced by 22.4%.

Decreased mir-45 expression activity exerts its anticardiomyocyte apoptosis effect by effectively reducing upregulated MIRI cardiomyocyte apoptosis and inhibiting cardiomyocyte activation of the AMPK signaling pathway. The AMPK signaling pathway has a good anti-inflammatory effect on the activation of endothelial cells. The activation of the AMPK signaling pathway effectively inhibits the mutual adhesion between the white blood cells and activated endothelial cells after endothelial ischemia and reduces the local endothelial cells caused by inflammation. Proliferation and aggregation can play a good anti-inflammatory effect. The results of the study found that miR-451 can reduce the inflammatory response of myocardial tissue during myocardial ischemia-reperfusion in rats by reducing the activity of AMPK signaling pathway. The specific data are shown in Figure 4.

It can be seen from Figure 4 that miR-451 can reduce the inflammatory response of myocardial tissue during myocardial ischemia-reperfusion in rats by reducing the activity of AMPK signaling pathway. When the expression level of miR-451 decreases by 15.7%, the inflammation of myocardial tissue during myocardial ischemia-reperfusion in rats is reduced. The response level was reduced by 33.6%.

With the rapid development of nanotechnology, more and more new nanomaterials have been used in the treatment of myocardial ischemia-reperfusion. Nanoceria pretreatment can upregulate the expression of Nrf2 in the reperfusion myocardium of rats, reduce the oxidative damage of reperfusion myocardium, and thus protect the myocardium. PBNP pretreatment can improve the ability of oxygen free radical scavenging and antilipid peroxidation of cardiomyocytes and reduce the apoptosis of cardiomyocytes. PAMAM-D nanocarrier can be used to carry AODN for gene therapy and has obvious preventive and therapeutic effect on myocardial ischemia-reperfusion injury in rats.

## 5. Conclusions

1. Cardiovascular disease is the number one killer of humans in the 21st century. Myocardial infarction is the main cause of death in patients with cardiovascular disease. At present, the main method of treating cardiovascular disease is perfusion therapy. Myocardial ischemia and reperfusion will inevitably cause reperfusion injury. This is also a major problem in the treatment of cardiovascular diseases. It is reported that miR-451 in the microRNA family participates in the protection of myocardial ischemia and reperfusion by regulating the myocardial adenylate-activated kinase AMPK. This article is based on this study
2. The results of the study showed that when the expression level of miR-451 was reduced by 15.7%, the activity index of AMPK signaling pathway increased by 18.3%, the area of myocardial infarction in rats was reduced by 22.4%, and the apoptosis rate of myocardial cells was reduced by 25.2%. The structure is improved. Therefore, it can be seen that miR-451 is an AMPK signaling pathway inhibitory gene. Decreasing the expression of miR-451 will increase the AMPK signaling pathway activity, and the increase in AMPK signaling pathway activity will help reduce myocardial ischemia-reperfusion injury
3. Studies have found that iR-451 improves myocardial injury during reperfusion in rats by regulating the activity of AMPK signaling pathway, enhances rat heart function, reduces the expression of positive cells in cardiomyocytes, and inhibits the proapoptotic factor. Caspase-3 at the same time, miR-451 can reduce the inflammatory response of myocardial tissue during myocardial ischemia-reperfusion in rats by reducing the activity of AMPK signaling pathway. When miR-451 expression level is reduced by 15.7%, the inflammatory response of myocardial tissue during myocardial ischemia-reperfusion in rats is reduced by 15.7%. The level was reduced by 33.6%

## Figures and Tables

**Figure 1:** The effect of downregulating the expression of miR-451 on the activity of AMPK signaling pathway.

**Figure 2:** The effect of miR-451 on the apoptosis rate of cardiomyocytes during ischemia-reperfusion by reducing the activity of AMPK signaling pathway.

**Figure 3:** The effect of miR-451 on the area of myocardial infarction during myocardial ischemia-reperfusion in rats by reducing the activity of AMPK signaling pathway.

**Figure 4:** The effect of miR-451 on the inflammatory response of myocardial tissue during myocardial ischemia-reperfusion in rats by reducing the activity of AMPK signaling pathway.

**Table 1:** Equipment and reagents used in this experiment.

Group	Usage amount	Source
Pipette	1	Beijing Zhuiqin Weise
1000 *μ*l sterile tip	2	Oxygen
50 ml centrifuge tube	2	Corning Corporation
CK-MB kit	270 ml	Caused by Jiangsu Feng Hua
RIPA Lysis Solution	320 mg	Merck Ka, Germany
Sodium chloride	280 ml	American SGH
Agarose	630 ml	American Sigma Company
Goat serum	400 ml	American KPL Company

**Table 2:** Rat left ventricular hemodynamic data after regulating the expression of miR-451.

Group	HR	LVDP	LVEDP	±DP/dt
I/R	252.3 ± 16	56.3 ± 5	13.6 ± 3	338.5 ± 25
DMSO	254.7 ± 15	60.4 ± 4	14.4 ± 4	366.4 ± 28
Downregulation group	237.2 ± 15	66.7 ± 5	12.5 ± 3	375.2 ± 19
Upregulation group	266.1 ± 17	57.7 ± 5	17.8 ± 5	342.9 ± 22

## Data Availability

All data available in this paper.
